# Repeated Low-Dose Streptozotocin and Alloxan Induced Long-Term and Stable Type 1 Diabetes Model in Beagle Dogs

**DOI:** 10.1155/2022/5422287

**Published:** 2022-08-08

**Authors:** Qingyue Han, Jie Sun, Wenting Xie, Yuman Bai, Shuzhou Wang, Jianjia Huang, Shuilian Zhou, Quanwei Li, Hui Zhang, Zhaoxin Tang

**Affiliations:** College of Veterinary Medicine, South China Agricultural University, Guangzhou, 510642 Guangdong, China

## Abstract

Type 1 diabetes mellitus (T1DM) is a chronic disease represented by insulin-causing pancreatic *β*-cell disruption and hyperglycemia. Therefore, it is necessary to establish a variety of animal models of diabetes to study the pathogenesis and pathophysiology of it. However, there are few reports on the use of beagle dogs to establish an animal model of type 1 diabetes. This study aimed to explore a simple and feasible modeling method to establish a long-term and stable type 1 diabetes model in beagle dogs. Forty adult beagle dogs were randomly divided into control group and model group. After 24 h of fasting, streptozotocin (20 mg/kg) and alloxan (20 mg/kg) were injected through the cephalic vein. The second intravenous injection was given on the 4th day after the first injection. Insulin release testing was performed on the 7th day after the last intravenous injection. Fasting blood glucose and body weight were recorded monthly. Four months after the last injection, the serum fructosamine content and the ratio of glycated hemoglobin were detected. Then, the pancreatic tissue was harvested for histopathological examination. The results showed that the level of fasting blood glucose of the 16 dogs in the model group was consistently higher than 11.1 mmol/L for 4 consecutive months. Moreover, compared with the control group, the insulin release curve of the model group was flat with no increase. The body weight of the model group was significantly reduced, and the ratios of blood glucose, fructosamine, and glycosylated hemoglobin were significantly higher than those in the control group. Meanwhile, histopathological examination of the pancreas showed that the islet beta cells appeared to have vacuoles or even necrosis. In the model group, pancreatic *β*-cells were damaged and insulin release was reduced. These results suggest that the above modeling methods can induce long-term and stable type 1 diabetes models in beagle dogs.

## 1. Introduction

Diabetes mellitus (DM) is a type of endocrine and metabolic disease whose etiology has not been fully elucidated. With the continuous in-depth research of DM, the experimental animals of DM models are not limited to small experimental animals such as mice and rabbits. Large mammal animal was used to establish a metabolic disease model because of its higher similarity to humans than other small animals [1, 2]. The advantage of using a large animal model is that its size, pancreas, and islet structures are similar to those of humans. It has similar physiological functions and pharmacokinetics to humans. Its long life cycle is more conducive to long-term research. The stress of large animals during the experiment can be relieved by training [1, 3]. Diabetes mel litus is one of the most common endocrine diseases affecting pet dog [4]. The vast majority of canine diabetes is insulin-dependent diabetes, which is similar to human type 1 diabetes and is a good animal model for human type 1 diabetes treatment research [5]. However, there are few methods to establish a beagle DM model [6–8]. The main reason is that model dosage is difficult to control, there is greater variation between dogs than in the small experimental animals, such as age, weight, hormones, and individual physical conditions. At present, streptozotocin (STZ) and/or alloxan (ALX) were mainly used in T1D modeling. The purpose of this study is to induce beagle T1D through the combined use of small doses of STZ and ALX in two times. The success rate and mortality of modeling, body weight (BW), fasting blood glucose (FBG), fructosamine (FUN), glycosylated hemoglobin (HbA1c) ratio, and other indicators were detected within four months after modeling.

## 2. Materials and Methods

### 2.1. Experimental Animals

Forty adult beagle dogs (aged 2-3 years old, half males and females, each weighing about 10 kg) were used in this study. After the dogs had been adaptively fed for 2 weeks in a controlled environment with a temperature of 22-25°C and relative humidity of 35%-50%, the experiment was conducted. This protocol was approved by the Animal Care and Use Committee of the Laboratory Animal Center of South China Agricultural University (ethics review certificate number: 2021A041).

### 2.2. Reagents and Main Instruments

STZ was purchased from Shanghai Yuanye Biotechnology Co., LTD.; ALX was purchased from Sigma, USA. Canine INS ELISA kit and canine glycosylated hemoglobin detection kit were purchased from Shanghai Zhen Ke Biological Technology Co., LTD.; Yuwell 586 blood glucose test strips and blood glucose meter and FUN detection reagent were purchased from Shenzhen Mindray Animal Medical Technology Co., LTD.; automatic biochemical analyzer was purchased from Mindray BS380; automatic blood cell analyzer was purchased from Mindray BC-5000 Vet; laser confocal microscope was purchased from TCS Sp8 Leica, Germany.

### 2.3. Preparation of Drug Solutions

The solvent of STZ is 0.1 mol/L citric acid buffer (pH = 4.5). The solvent of ALX is 0.9% saline. The configuration concentration of STZ and ALX is 5%.

### 2.4. Grouping and Modeling

Forty beagle dogs were randomly divided into two groups, twenty dogs for each group. Before injection, dogs were fasted for 24 h, and ear vein blood was taken to measure FBG. The STZ and ALX were put into their respective EP tubes, wrapped in aluminum foil (avoiding light), and stored on ice. The corresponding amount of solvent was extracted to dissolve the medicinal solution and shaken vigorously to ensure complete dissolution. The dogs were given a rapid intravenous injection in the dark room. The second dose was given on the fourth day (72 h later). The dosage and method of injection were the same as the first time. The control group was given the same amount of normal saline (NS) in the same way. The timeline of injections is shown in Figure 1.

### 2.5. Insulin Release Test (IRT)

On the seventh day after the second injection, dogs in both groups were orally administered 10 mL/kg of 50% high glucose solution on an empty stomach. Blood was collected before and 0.5, 1, 2, and 3 hours after feeding, and the serum was obtained to detect the insulin levels.

### 2.6. Fasting Blood Glucose (FBG) and Body Weight (BW)

FBG and BW were measured monthly after four months of the injection. The dog's diet, water intake, and physical and mental state were observed and recorded during this period.

### 2.7. Fructosamine (FUN) and Glycosylated Hemoglobin (HbA1c)

After 4 months of injection, fasting blood was collected to detect the contents of FUN, hemoglobin (HGB), and HbA1c. The HbA1c ratio was calculated.

### 2.8. Histopathological Examination of the Pancreas

Four months after injection, the experimental dogs were sacrificed after anesthesia, and the pancreatic tissue was collected, fixed, dehydrated, embedded, and then stained with hematoxylin-eosin (HE). Histopathological changes were observed under a microscope and photographed.

### 2.9. Statistics

The results were expressed as mean ± standard error of the mean (SEM). GraphPad Prism 9 (GraphPad Inc., USA) was used for the visualization of graphs and data analysis. Differences were evaluated by using one-way ANOVA. *P* < 0.05 indicates that a difference is statistically significant (^∗^*P* < 0.05, ^∗∗^*P* < 0.01, ^∗∗∗^*P* < 0.001, or ^∗∗∗∗^*P* < 0.0001).

## 3. Results

### 3.1. General Observation

After the first injection, the dog developed depression, curled up, and had decreased appetite. After 15-24 h, dogs vomited pale yellow foamy mucus. After the second injection, some dogs still had vomiting, while other adverse symptoms were significantly reduced compared with the first injection. One week after the injection, the dogs' state was stable, and the appetite recovered. The model dogs were depressed, decreased in activity, increased in diet and drinking, and increased in urine in 2-4 months. The control group behaved normally. After the injection, two dogs in the model group showed a significant increase in serum liver and kidney biochemical indicators. They did not drink or eat and died in one week after modeling. Necropsy revealed that the liver and kidney organs were seriously damaged, and the gallbladder was necrotic. Another dog that did not eat or drink received 200 mL of 5% dextrose saline intravenously every day and died on the 10^th^ day after modeling. Anatomical examination showed diffuse hemorrhage of internal organs. There was another dog in a special situation whose FBG was always in the normal range after several injections. The modeling success rate is 80%.

### 3.2. Insulin Release Test

After feeding glucose solution, the insulin release level of the model group was low and with no peak. In the control group, the release curve showed a trend of rising at first and then falling, with a peak at 0.5 h. The results of the IRT between the two groups are significantly different (Figure 2). The results showed that the model's type is type 1 diabetes.

### 3.3. FBG and BW Changes

Four months after the injection, the FBG levels of the two groups of dogs were detected. The results showed that the level of FBG in the model group was significantly higher than that of the control group (*P* < 0.0001, Figure 3). Moreover, the results showed that compared with the control group, the weight of the model group decreased significantly (*P* < 0.0001, Figure 4). Dogs in the model group experienced progressive weight loss (Figure 5). In the model group, the ribs of the dogs became visible, the waist and pelvis were clearly defined. Compared with the control group, the muscle and fat contents of the model group reduced significantly.

### 3.4. FUN and HbA1c Changes

FUN was significantly increased in the model group compared with the control group (*P* < 0.01, Figure 6). Furthermore, the percentage of HbA1c increased in the model group and the results were significantly different compared with the control group (*P* < 0.05, Figure 7).

### 3.5. Histomorphological Examination of Pancreas

The results of histopathology experiments of the pancreas showed that compared with the control group, the islets of the pancreas in the model group were severely damaged (Figure 8). Main changes were as follows: (1) the area of the islets has become smaller, and there are even only narrow and long remnants formed by a few cells (the yellow arrow indication). (2) Pancreatic islet cells (mainly *β*-cells) decrease (atrophy), and the remaining cells are vacuolated or even necrotic (the red arrow indication). (3) The exocrine gland cells can be degenerated (the black arrow indication).

## 4. Discussion

As we all know, DM is a research hotspot in the field of scientific research. At present, there are many studies on small diabetic animal models such as rats, rabbits, and hamsters, and the modeling technology has been relatively mature, but there are few studies on large diabetic animal models such as dogs [7–9]. The small diabetic animal models are widely used in the research and development of diabetes drugs or technologies, but with the limitations of body size and lifespan, it has limited reference significance for the clinical treatment of diabetes [10]. Beagle dogs with stable genetic performance, fixed and excellent breed, and generally free from hereditary neurological disorders are internationally recognized as a model for experiment. Thus, it would be useful to establish a beagle dog model of diabetes for the study of the pathogenesis and pathophysiology of diabetes.

Both STZ and ALX can selectively destroy pancreatic *β*-cells through their toxic effects, inducing a chronic DM state [6, 11, 12]. Alloxan is far less expensive and more readily available than streptozotocin. STZ has longer half-life (15 min against 1.5 min of alloxan) [13]. This makes it more stable in solution before and after injection into animals. STZ-induced hyperglycemia is relatively more stable and for a longer duration. Moreover, the mechanism of STZ diabetogenicity is less associated with cellular toxicity and lesser animal mortality [14]. The combination of STZ and ALX can reduce the dose than using both alone, which can reduce the hepatic and renal damage [7, 14].

Black et al. used ALX (50 mg/kg) and STZ (30 mg/kg) and concluded that dogs with high BW had significant hepatic and renal injury and increased mortality [6]. Anderson et al. used ALX (40 mg/kg) and STZ (35 mg/kg) which were administered, and the modeling failure rate was 12.5% [15]. In addition, Salis et al. induced canine DM by infusing ALX (20-25 mg/kg) and STZ (20-25 mg/kg) in the suprarenal artery during pararenal abdominal aortic balloon occlusion [16]. This modeling method increases the modeling procedure time compared to intravenous injection and increased modeling costs. The blood glucose of dogs reached the nadir 12-16 h after injection, which was caused by severe hypoglycemia caused by the release of insulin from damaged *β*-cells. When the nadir blood glucose is below 3.0 mmol/L, the dog is given 0.5 mL/kg of 50% high glucose solution via the cephalic vein in the forelimb to relieve the dog's hypoglycemic state, maintain the vital signs, and avoid death caused by transient hypoglycemia. Appetite was affected in some dogs. Two days after the end of the modeling injection, when the dog had poor appetite, we adjusted the food composition (feeding canine ham, milk, chicken breast puree, etc.) to induce the dog's appetite to return. When the diet was less for more than 3 days, 5% glucose saline was intravenously injected to maintain the body's energy metabolism. In order to improve the reproducibility of the modeling method, we did not do much to interfere or rescue the dog. The experimental results showed that the success rate of the modeling method in this study was 80%, the mortality rate was 15%, and the failure rate was 5%. This indicates that the small-dose multiple injection methods reduced the damage of the modeling drug to the dogs and improved the model success rate.

The criteria for the onset of DM were the presence of DM symptoms and a random plasma glucose concentration ≥ 11.1 mmol/L or fasting plasma glucose concentration ≥ 7.0 mmol/L or OGTT 2 h plasma glucose concentration ≥ 11.1 mmol [17]. Dogs are considered diabetic if the blood glucose is higher than 11.1 mmol/L for two consecutive weeks. Insulin release test can reflect the functional status of pancreatic beta cells and guide treatment. IRT in this experiment showed that the curve of the model group was low and flat, and the insulin production value decreased, indicating a decrease in insulin synthesis and secretion. This study enriches the scientific detection method of canine DM model typing. It was shown that pancreatic cells modeled with the combination of two drugs showed nuclear chromatin clumps, vacuolation of mitochondria, and enlargement of the endoplasmic reticulum unilateral map. The secretory granules appeared swollen. Cell degeneration was severe. *α* and *δ* cells seemed unaffected. This experiment showed that pathomorphological section staining of the pancreas four months after modeling showed severe damage and lesions in the islet region of the pancreas in the model group. The islet region of the model group of dogs was damaged, and the *β*-cells have degenerated and are necrotic. It is evident that irreversible damage to the pancreas occurred after the injection of the drug, and the damage lasted for 4 months.

## 5. Conclusions

In summary, we can conclude that the model group of dogs has become a long-term and stable T1D model. The method of chemically inducing the T1D model in dogs with a small number of combined doses is safe, simple, and reliable and has a high modeling rate. It is a more ideal method for inducing the T1D model in large animals and has good implications for future diabetes research.

## Figures and Tables

**Figure 1:** The timeline of injections.

**Figure 2:** Insulin release levels before and 0.5, 1, 2, and 3 h after feeding.

**Figure 3:** Fasting plasma glucose levels of groups.

**Figure 4:** Body weight changes of groups.

**Figure 5:** Posture and body shape observation of dogs. After 4 months of rearing and modeling, the dogs were photographed before being sacrificed. C1-C3 are the pictures of 3 dogs randomly selected from the control group. M1-M3 are the photos of 3 dogs randomly selected from the model group.

**Figure 6:** Fructosamine levels of groups.

**Figure 7:** Percentage of HbA1c of groups.

**Figure 8:** HE staining of pancreas tissue. The yellow arrows indicate islet regions, the red arrows indicate damaged islet cells, and the black arrows indicate exocrine ducts. No ketoacidosis occurred in all dogs during the experiment.

## Data Availability

The data that support the findings of this study are available from the corresponding author upon reasonable request.
